The article "Sustainable Development of Green Reverse Logistics Based on Blockchain" was retracted in 2023. Reasons: signs of a paper mill; suspected computer-generated content; unreliable results or conclusions; lack of ethics approval or compliance.

# Sustainable Development of Green Reverse Logistics Based on Blockchain

**DOI:** 10.1155/2022/3797765

**Published:** 2022-09-02

**Authors:** Zhiqi Wu, Zhiqi Zhao

**Affiliations:** School of Economics and Management, Zhengzhou Normal University, ZhengZhou 450044, Henan, China

## Abstract

With the depletion of global resources and the deterioration of the ecological environment, the implementation of green reverse logistics management has become a necessary means. Green reverse logistics is a new type of reverse logistics that aims to improve resource utilization and protect the ecological environment. While promoting sustainable development, “green reverse logistics” also has certain social and economic significance. This paper compared the green reverse logistics system based on blockchain with the current green reverse logistics system. Taking drug recycling as an example, this paper mainly analyzed the waste rate, utilization rate, and enterprise income. The comparison results showed that the efficiency of drug recycling based on blockchain has increased by 20.1% compared with the current stage, and the waste rate has decreased by 16%. The utilization rate has increased by 14%, and corporate income has also increased by 19.5%. It is greatly indicated that green reverse logistics based on blockchain is of great significance to enterprise income and environmental protection, which also produces great social benefits.

## 1. Introduction

The rise of green reverse logistics stems from people's widespread concern about environmental issues. After the Second World War, the rapid development of the world's productive forces also had a serious impact on the Earth's ecological environment, including the poorer quality of the world's environment, unclean air quality, widespread industrial waste, waste products, and so on. The massive consumption of resources has a great impact on human life and economic development.

The best way to realize green reverse logistics is through recycling and reproduction. It is a recyclable regeneration system that can fully recycle various renewable resources and can also reduce the disposal cost of waste, thereby obtaining huge economic benefits. In addition, due to the reduction in the amount of garbage, the pollution to the environment is also reduced, and the ecological environment is protected, thereby promoting ecological balance. Reverse logistics is a system of utilization, remanufacturing, and recycling. It can not only make full use of resources but also effectively protect the ecological environment, which brings great economic and social benefits.

In this paper, by comparing the current reverse logistics with the green reverse logistics based on blockchain, it was found that the recycling efficiency of green reverse logistics based on blockchain has increased significantly from 61.3% to 81.4%. In terms of abandonment rate and utilization rate, the abandonment rate has been effectively reduced. The utilization rate has been significantly improved, and corporate income has also been improved.

The article "Sustainable Development of Green Reverse Logistics Based on Blockchain" was retracted in 2023. Reasons: signs of a paper mill; suspected computer-generated content; unreliable results or conclusions; lack of ethics approval or compliance.

## 2. Related Work

Global technology continues to develop, but nonrenewable energy sources are becoming less and less, which makes people begin to pay attention to sustainable development. Feris tried to make good management decisions at the environmental level. He understood and explained the relationship between environmental management and sustainable development in South Africa. The report critiqued recent cases and sought to understand how Chinese courts evaluate environmental decision-making [1]. Multinational corporations play a pivotal role in achieving the sustainable development goals. Kolk et al. explored their behavior in implementing SDGs. He reviewed the positive and negative impacts of human beings on the prosperity and peace of the Earth as determined by the United Nations 2030 Agenda and summarized 61 related research results. The result was that the number of positive impacts is greater than the number of negative impacts, but the negative impacts may bring about insecurity on the Earth [2]. Sustainability issues are increasingly the focus of global organizations and stakeholders. In this context, eco-efficiency has become a means of constant transformation into sustainable development. Caiado et al. systematically reviewed sustainable development issues from the perspective of eco-efficiency and used knowledge of the knowledge development process to identify and construct the latest eco-efficiency and sustainable development technologies. A statistical analysis of the selected BPs was carried out, and a thematic synthesis was carried out, combining ecological benefits and sustainable development with other approaches [3]. Plessis and Rautenbach offered several legal perspectives on sustainable development issues. Taking sustainable development as an environmental concept, in the living space, a specific concept and culture can be better integrated into the formula of sustainable development. The study found that in the context of sustainable development, the fluidity and importance of culture need to be differentiated from the role of culture and the role played in sustainable development [4]. The issue of sustainable development has attracted the attention of scholars around the world. In sustainable development, some of them have discussed the issue of green reverse logistics.

The article "Sustainable Development of Green Reverse Logistics Based on Blockchain" was retracted in 2023. Reasons: signs of a paper mill; suspected computer-generated content; unreliable results or conclusions; lack of ethics approval or compliance.

In terms of green reverse logistics, many scholars have discussed it. Due to the shortage of resources, air and environmental pollution and the sustainable development of the environment has become a common concern of people. The logistics industry has added green logistics concepts and functions such as green logistics and reverse logistics. The purpose of Ali et al. was to understand the drivers and obstacles of reverse logistics and to analyze the impact of reverse logistics in terms of time, cost, technology, and green concept [5]. Diversified design and production have played a significant role in reducing the amount of electronic waste in waste electronic products. A green supply chain management framework combines environmentally friendly practices with sustainable production and consumption. Khor et al. explored eco-design, reverse logistics, demolition design, and business performance (eco-efficiency and profit). Using the variance structure equation model, the survey data of 89 electric power and electronic enterprises that have obtained IS014001 certificates were analyzed. The research results showed that the disassembly design has a certain impact on the environmental design and has a certain impact on the realization of reverse logistics. Further research found that reverse logistics has a significant relationship with environmental benefits and profits, but the ecological design did not bring similar effects [6]. With the negative effect of environmental pollution, environmental sensitive issues have become increasingly prominent. To achieve a sustainable life, people's production and lives must adapt to the environment. In this context, Yldz and Avdar studied the impact of reverse logistics on environmental and economic performance. The data were surveyed by 191 production enterprises. The collected data were analyzed using structural equation modeling and the macroprocess method. Using structural equation modeling, the significant impact of green production on environmental and economic performance was studied [7]. Relevant scholars have conducted research on the issue of sustainable development but not under the blockchain technology. In this regard, this paper discusses the sustainable development of green reverse logistics based on blockchain.

## 3. Green Reverse Logistics

### 3.1. Significance of Sustainable Development of Green Reverse Logistics

Minimizing waste can achieve sustainable development [8]. Waste management is generally aimed at reducing residues in industrial production, and there are two ways to reduce waste generation. One is to “turn waste into treasure” for existing garbage, and the other is to recycle it. The specific methods are a reduction in the amount of waste and recycling of waste. Generally speaking, the best way is to use the waste generated by resources as much as possible and try to avoid the generation of waste in one place. If garbage has already been created, then it needs to be sure to maximize its meaning, preferably reusing it. If not, it should be recycled. In order to maximize the utilization of resources, it has laid the foundation for the sustainable development of resources. At the same time, achieving the balance of material and energy ecology will be the development trend of China's industrial manufacturing.

The article "Sustainable Development of Green Reverse Logistics Based on Blockchain" was retracted in 2023. Reasons: signs of a paper mill; suspected computer-generated content; unreliable results or conclusions; lack of ethics approval or compliance.

Good management of reverse logistics can promote the sustainable development of the economy [9]. Among the many activities of reverse logistics, the most important is the management of customer returns. For reverse logistics in the field of circulation, the following methods can be taken to reduce the amount of commodity recycling as much as possible. First, a recycling logistics system can be established in the whole supply chain. The management of reverse logistics should start by preventing the backwardness (that is, returning) of products. As long as the logistics company can make strategic demands on each employee, it can prevent (or reduce) the backwardness of certain products. Second, it is necessary to establish the disassembly-oriented design idea. That is, in the design of the product, the reprocessing and reuse of the product should be fully considered.

The reverse development of green logistics [10]: The greening of reverse logistics can be started from two aspects. One is the green reuse of waste, and the other is environmental protection. In other words, the recycling of waste products is an environmentally friendly behavior. If the whole world is one-way, then the domestic waste of producers and consumers will spread to the entire planet in a short period of time, causing unimaginable environmental pollution and waste of resources. Generally speaking, the best way for the green development of renewable logistics is recycling and reproduction. It is a renewable material that can effectively recover various useful resources and reduce the disposal cost of waste, thereby achieving high economic benefits. In addition, due to the reduction in the amount of garbage, the pollution to the environment is reduced, so that the ecological environment can be maintained. This creates a broad development space for the sustainable development of the enterprise and realizes the strategic goal of sustainable development of the enterprise. The significance of the sustainable development of green reverse logistics mainly lies in the aforementioned three points: minimizing waste, managing reverse logistics, and the reverse development of green logistics, as shown in Figure 1.

The article "Sustainable Development of Green Reverse Logistics Based on Blockchain" was retracted in 2023. Reasons: signs of a paper mill; suspected computer-generated content; unreliable results or conclusions; lack of ethics approval or compliance.

### 3.2. Development Strategy of Green Reverse Logistics under the Concept of Sustainable Development

Taking green reverse logistics is an important way to achieve sustainable development, as shown in Figure 2. The sustainable development of society is inseparable from the strong support of society. Therefore, it is necessary to strengthen the social awareness of environmental protection and resource conservation and establish the concept of sustainable development. The government should change its attitude of emphasizing economic development, ignoring the ecological environment, economic benefits, social benefits, immediate interests, and long-term interests. Instead, it should establish resource and environmental awareness and adhere to the strategy of sustainable development [11].

As the main body of the implementation of reverse logistics, enterprises should start from the perspective of sustainable development, attach importance to the operation of reverse logistics, and raise reverse logistics to the level of an enterprise development strategy. At the same time, people must pay attention to the research and development and design of products to make them more environmentally friendly and easier to recycle. It is also necessary to strengthen the control of the production process and strictly check to minimize the problems of products entering the market caused by improper production management, thereby reducing the return caused by product quality problems. Through the introduction of reverse logistics, enterprises can effectively reduce the waste of resources and reduce environmental pollution. Consumers should start with the concept of sustainable development and advocate “green” reverse logistics [12]. For example, people can replace plastic bags with vegetable baskets as much as possible, consume simple packaged food, and reduce disposable consumer goods. It is necessary to understand the grading standards of waste disposal and to divide waste into recyclable and nonrecyclable to facilitate reuse. Household appliances, computers, and other durable goods can be recycled by way of “trade-in.” In addition, consumers themselves should not only engage in green consumption but also actively participate in the recycling of renewable resources and environmental protection. They can vigorously promote the concept of resource recycling and green consumption in society, advocate the behavior of green reverse logistics, and supervise the government to strengthen reverse logistics management. There are three main factors to achieving green reverse logistics, as shown in Figure 3.

The article "Sustainable Development of Green Reverse Logistics Based on Blockchain" was retracted in 2023. Reasons: signs of a paper mill; suspected computer-generated content; unreliable results or conclusions; lack of ethics approval or compliance.

Technology is the key to realizing green reverse logistics [13]. It is necessary to strengthen green technical support to ensure the production process has green logistics. At present, domestic waste recycling, disposal, and recycling technology is relatively backward. The cost of reverse logistics is high, and the utilization rate of renewable resources is not high. Because much waste cannot be recycled and processed due to technical reasons, it directly enters the ecological and social system, causing serious environmental pollution. Therefore, technical problems have become a “bottleneck”, hindering the development of reverse logistics in China. At present, while actively promoting independent innovation, China should also strengthen research on technologies related to reverse logistics, as shown in Table 1. There are three main aspects: improving quality, strengthening recycling technology, and creating energy-saving technologies. First, enterprises should be encouraged to improve product design, improve product quality, green production, promote green packaging, and secure the door to “reverse logistics.” Second, the development of recycling technology determines the way and method of recycling. Third, creating technologies such as new energy-saving technologies, clean energy, and environmentally friendly vehicles has positive significance for improving energy consumption and exhaust emissions in the logistics process.

Strengthening informatization [14]: The uncertainty and complexity of reverse logistics can be seen from the operation mode of reverse logistics. In the process of reverse logistics, there is uncertainty about the information on the recovery and reprocessing of the product. For example, product composition, recycling quantities, remanufactured parts, and material requirements, product recycling processing operations, etc., are all unclear. To a certain extent, the informatization of reverse logistics is more important than forward logistics. Therefore, strengthening information construction and building a reverse logistics information network can help enterprises understand the operation status of reverse logistics in a timely manner and enhance their enthusiasm for participating in reverse logistics. First, reverse logistics uses advanced information technology. The basic information of the product (basic product information, quality status, the reason for return, etc.) can be effectively tracked, for example, using barcode technology. Second, the use of advanced modern logistics information networks, such as GPS and network technology, can effectively track and manage the entire process of reverse logistics. It greatly reduces the processing time of logistics, which is conducive to optimizing the optimal design of the logistics system, optimizing the sharing of logistics resources, and reducing ineffective logistics, which will reduce energy consumption and pollution, thus realizing the greenness of the logistics process.

The article "Sustainable Development of Green Reverse Logistics Based on Blockchain" was retracted in 2023. Reasons: signs of a paper mill; suspected computer-generated content; unreliable results or conclusions; lack of ethics approval or compliance.

Choosing an appropriate way for the development of reverse logistics [15]: From the perspective of a logistics organization, there are three main logistics methods: One is the company that produces the waste to carry out the logistics. Another is the company that needs the waste to operate and recycle the required waste. The third is the reverse logistics of the third party. At present, the development of reverse logistics is still in its infancy, and the market for reverse logistics is not yet fully mature. Enterprises should conduct comprehensive thinking and decision-making from the perspectives of enterprise scale, strength, reverse logistics cost, reverse logistics technology, and reverse logistics capabilities. Generally, products with a high unit value are recycled, such as waste copiers, electrical assembly products, etc. After reprocessing or assembly, these products can be reused for high profit. At the same time, the company will also consider the confidentiality of core technologies as well as the impact of the recycling network on the company's reputation and brand. For enterprises with lower unit value but higher requirements for postrecycling processing equipment and processes, higher processing costs, smaller scale, and less capital, they usually cannot complete recycling. They take the second way of operating independently, or the government appoints professional institutions to undertake it. For processing equipment with a certain scale economy value, packaging materials with simple processes, wine bottles, and so on, a third-party logistics company can be entrusted for distribution. This is mainly due to the professional logistics network, advanced logistics management system, and professional management level of third-party logistics enterprises, which can determine the reverse logistics and how to carry out logistics activities according to specific enterprises and can collect, classify, and process recycled products in a centralized manner to achieve economies of scale. Second, it can provide a relatively complete reverse logistics management system for third-party logistics enterprises without spending time and costs. The supply and demand sides of reverse logistics can establish a strategic partnership through contracts and determine the allocation of their costs, benefits, and risks so as to achieve the purpose of risk sharing and benefit sharing. Third, in order to enhance the company's competitiveness, it can concentrate its strength and resources on developing its own core business.

The article "Sustainable Development of Green Reverse Logistics Based on Blockchain" was retracted in 2023. Reasons: signs of a paper mill; suspected computer-generated content; unreliable results or conclusions; lack of ethics approval or compliance.

### 3.3. Reverse Logistics of Drug Recall Based on Blockchain

In fact, the blockchain is a distributed system. It is a group of computers with independent functions. They cooperate with each other to complete a common task, but in the eyes of the end user, it is like a computer [16]. Blockchains have more and more records that are controlled by multiple entities that do not trust each other. Data is allocated to a block in batches or blocks. Each block contains the cryptographic hash of the previous block, which embeds the secure representation of the existing block into the block. Blockchain is a distributed system, and its consistency depends on FLP and CAP. In a distributed system, it is best to satisfy two of the three conditions of consistency, availability, and partition fault tolerance [17]. Typically, consensus algorithms in blockchains assume three roles, which are proposer, receiver, and executor.

1. Adviser: it usually refers to the leader whose role is to propose.
2. Recipient: it hears the request for a proposal and provides a response.
3. Executor: it refers to other processes that accept the final decision in the system.

If the following conditions are met, it can be called “distributed consistency.” If the conditions are not met, it will be output directly at that corresponding stage. The first is consistency. That is, all nodes that have not failed will choose the same output. The second is the end. All fault-free nodes will choose an output that cannot exit. The third is completeness. If all nodes give the same value, the value is finally output by the system.

This article illustrates the problem of drug recovery in reverse logistics. For a long time, China has not paid enough attention to the reverse logistics of medicine, and most expired medicines are discarded or thrown directly into the trash can. This not only causes great waste but also has a great impact on human health. At present, scholars at home and abroad have discussed the related issues of reverse logistics, but they mainly focus on the connotation and causes of reverse logistics while ignoring the application of information technology in pharmaceutical reverse logistics [18]. The whole process of reverse logistics of drug recovery can be summarized into four major links mainly including collection, statistics, transportation, and processing, as shown in Figure 4.

According to the randomness of drug quality, a network model of point-of-sale for drug sales is established, as shown in Figure 5. The center is a point-of-sale for drugs In order to facilitate the collection and analysis of drugs, data is collected by suppliers and then distributed to various distribution centers [19], so that the collection and processing centers are centralized and equipped with special personnel and equipment, which saves transportation costs, reduces warehouse management costs, and improves space utilization.

The article "Sustainable Development of Green Reverse Logistics Based on Blockchain" was retracted in 2023. Reasons: signs of a paper mill; suspected computer-generated content; unreliable results or conclusions; lack of ethics approval or compliance.

At retail locations, problematic drugs are sent to a centralized location where there are no capacity constraints, and the quality of the drugs can also be detected and then transported through different transportation nodes to the drug company's recycling depot. In this process, each node has a limit [20]. These stages are modeled and described below.

From the retail point to the recycling center [21], at this stage, the distribution fee is only related to the distribution distance. After the distribution center gives a certain rebate reward to the distribution point, the retail point will distribute it to the third-party logistics center, and the distribution center will conduct inspection and classification. Its tariff function is as follows:

(1) $$\begin{array}{c} W_{0}=B_{ij}c_{0ij}. \end{array}$$

From recycling center to transport node [22]; in the investigation, three different situations can be classified according to the severity of the product quality defect: severity of product quality (category I); the severity of product quality (category II); the severity of product quality (category III). If the product quality problem severity value is (0, S2), then the product belongs to category III. If the product's quality problem severity is (S2, S1), then the product belongs to category II. Medicines in the primary and secondary categories are put on the mandatory recall list. Therefore, for different problematic drugs, the transportation measures taken are different, so the required unit distance transportation costs are also different. Because the recycling machine collection area can detect the defects of medicines, the numbers of medicines with different defect grades at each collection point are as follows:

(2) $$\begin{array}{c} Q_{i1}=\int_{S_{1}}^{1}\sum_{j}c_{ij}f\left(S_{1i}\right)\text{d}S_{1i}, \end{array}$$

(3) $$\begin{array}{c} Q_{i2}=\int_{S_{2}}^{S_{1}}\sum_{j}c_{ij}f\left(S_{1i}\right)\text{d}S_{1i}, \end{array}$$

(4) $$\begin{array}{c} Q_{i3}=\int_{0}^{S_{2}}\sum_{j}c_{ij}f\left(S_{1i}\right)\text{d}S_{1i}. \end{array}$$

The single-cycle transportation cost function at this stage is as follows:

(5) $$\begin{array}{c} W_{1}=\sum_{i,m}x_{im}p_{k}d_{1im}d_{1im}\left(\int_{S_{1}}^{1}p_{1}f\left(S_{1i}\right)\text{d}S_{1i}\right)+\int_{S_{2}}^{S_{1}}p_{2}f\left(S_{1i}\right)\text{d}S_{1i}+\int_{0}^{S_{2}}p_{3}f\left(S_{1i}\right)\text{d}S_{1i}. \end{array}$$

The conditions that need to be met are as follows:

(6) $$\begin{array}{c} \sum_{m}\int_{S_{1}}^{1}x_{im}f\left(S_{1i}\right)\text{d}S_{1i}\leq Q_{i1}, \end{array}$$

(7) $$\begin{array}{c} \sum_{m}\int_{S_{2}}^{S_{1}}x_{im}f\left(S_{1i}\right)\text{d}S_{1i}\leq Q_{i2}, \end{array}$$

(8) $$\begin{array}{c} \sum_{m}\int_{0}^{S_{2}}x_{im}f\left(S_{1i}\right)\text{d}S_{1i}\leq Q_{i3}, \end{array}$$

(9) $$\begin{array}{c} \sum_{m}x_{im}a_{1im}j_{1im}=T_{m}^{1}\leq c_{m}. \end{array}$$

Transport between transport nodes [23]: considering the influence of the defect degree of the medicine on the transportation cost, it is necessary to calculate the current storage capacity of the defective medicine at each node, as shown in the following equation:

(10) $$\begin{array}{c} T_{m}^{1}=\sum_{i}x_{im}a_{1im}j_{1im}. \end{array}$$

The transportation volume matrix between each transportation node is *X*_*mm*_, and its single-cycle transportation cost function is as follows:

(11) $$\begin{array}{c} W_{2}=\sum_{i,j}x_{ij}d_{2ij}a_{2ij}j_{2ij}\left(\int_{S_{1}}^{1}p_{1}f\left(S_{2i}\right)\text{d}S_{2i}+\int_{S_{2}}^{S_{1}}p_{2}f\left(S_{2i}\right)\text{d}S_{2i}+\int_{0}^{S_{2}}p_{3}f\left(S_{2i}\right)\text{d}S_{2i}\right). \end{array}$$

The conditions that need to be met are shown in the following equations:

(12) $$\begin{array}{c} \sum_{j}x_{ij}d_{2ij}a_{2ij}j_{2ij}\leq T_{i}^{1}, \end{array}$$

(13) $$\begin{array}{c} \sum_{i}x_{ij}d_{2ij}a_{2ij}j_{2ij}-\sum_{i}x_{ji}d_{2ji}a_{2ji}j_{2ji}+T_{j}^{1}\leq c_{j}. \end{array}$$

After the second stage, the current storage capacity of various types of defective drugs at each node is calculated, as shown in the following equation:

(14) $$\begin{array}{c} T_{m}^{2}=\sum_{i}x_{im}d_{2im}a_{2ij}j_{2ij}-\sum_{i}x_{mi}d_{2mi}a_{2mi}j_{2mi}. \end{array}$$

From hipping node to drug manufacturer recycling processing node: similar to the third stage, the transportation cost function of this stage is as follows:

(15) $$\begin{array}{c} W_{3}=\sum_{m,t}x_{mt}d_{3mt}a_{3mt}j_{3mt}\left(\int_{S_{1}}^{1}p_{1}f\left(S_{3i}\right)\text{d}S_{3i}+\int_{S_{2}}^{S_{1}}p_{2}f\left(S_{3i}\right)\text{d}S_{3i}+\int_{0}^{S_{2}}p_{3}f\left(S_{3i}\right)\text{d}S_{3i}\right). \end{array}$$

The conditions that are met are shown in the following equations:

(16) $$\begin{array}{c} \sum_{t}x_{mt}d_{3mt}a_{3mt}j_{3mt}\leq T_{m}^{2}, \end{array}$$

(17) $$\begin{array}{c} \sum_{m}x_{mt}d_{3mt}a_{3mt}j_{3mt}\leq ce_{t}. \end{array}$$

After the end of the previous stage, the storage capacity of various types of defective drugs at each node is calculated, as shown in the following equation:

(18) $$\begin{array}{c} T_{m}^{3}=T_{mk}^{2}-\sum_{t}x_{mt}d_{3mt}a_{3mt}j_{3mt}. \end{array}$$

Modeling the total transportation cost: the transportation cost of the i-th cycle is the sum of the transportation costs of each stage, as shown in the following equation:

(19) $$\begin{array}{c} W_{i}=W_{0}+W_{1}+W_{2}+W_{3}. \end{array}$$

The main function of the logistics system is to minimize cost. This mode can ensure that medicines in each logistics node in the network can only be delivered or directly delivered to the recycling station of the pharmaceutical company. Thus, it is ensured that the recycling station of the pharmaceutical supplier becomes the final receiving point, so as to ensure that all the medicines in the secondary cycle can reach the collection point.

The article "Sustainable Development of Green Reverse Logistics Based on Blockchain" was retracted in 2023. Reasons: signs of a paper mill; suspected computer-generated content; unreliable results or conclusions; lack of ethics approval or compliance.

The number of loops *n*=*n*_1_+*n*_2_+…*n*_*q*_, where q is the number of times to adjust the parameters of a single loop. The total transportation cost function is as follows:

(20) $$\begin{array}{c} W_{\text{total}}=\sum_{i}^{q}n_{i}W_{i}. \end{array}$$

Solving this equation by a final calculation yields the desired value.

## 4. Comparison of Blockchain-Based Green Reverse Logistics

In this paper, a data query is carried out on the amount of drug recovery in several regions. In order to verify the accuracy of the data, the recovery of some pharmaceutical companies in daily medicine was investigated. Through questionnaires, the recovery time and cost of recovery, as well as the number of local drug sites, could be learned. Through mathematical verification, it was found that the survey data was in line with the online data. Through the analysis of the data from the drug website, the reverse logistics of drug recycling not based on blockchain (represented by reverse logistics at the current stage in the following text) and the reverse logistics based on blockchain (represented by C and Q in Figure 6) were analyzed in four aspects: enterprise recycling efficiency, abandonment rate, utilization rate, and enterprise income.

The recycling efficiency of enterprises is mainly related to the transmission between nodes. At this stage, there are deficiencies in reverse logistics in drug recovery, and there is no uniformity, resulting in relatively low recovery efficiency. The recycling efficiency of enterprises based on blockchain will be relatively better. The blockchain can achieve regular node information transmission in each link so as to achieve relatively high recycling efficiency. In the two quarters, the comparison of recovery efficiency between the two is shown in Figure 6.

The article "Sustainable Development of Green Reverse Logistics Based on Blockchain" was retracted in 2023. Reasons: signs of a paper mill; suspected computer-generated content; unreliable results or conclusions; lack of ethics approval or compliance.

From the comparison of Figure 6, it can be found that the recovery efficiency of drugs at this stage was only about 61.3%, while the recovery efficiency based on blockchain has reached 81.4%. Compared with the current stage, the recovery efficiency has increased by 20.1%, which shows that blockchain-based drug recovery is more effective.

The abandonment rate refers to the ratio of drugs that fail to meet the recycling requirements of all recycled drugs. This index can also be used to judge the sustainable development of enterprises. Utilization is the ratio of the amount people use to the total output of all drugs after they are sold. They are all important indicators for judging whether a company is pursuing sustainable development or not. The comparison between the current reverse logistics and blockchain-based reverse logistics in terms of waste rate and utilization rate is shown in Figures 7 and 8.

Through two sets of data, it could be found that the current abandonment rate of reverse logistics was between 22% and 28%, and the utilization rate was between 75% and 79%. The abandonment rate based on blockchain was between 7% and 11%, and the utilization rate was between 87% and 95%. The reduction in the waste rate and the improvement of the utilization rate showed that reverse recycling based on the blockchain is conducive to sustainable development, which can reduce the waste of medicines and reduce the damage to the environment.

The main purpose of pharmaceutical companies is to make profits, and cost control is an important part of that. It is related to the survival of the enterprise. Through the recycling of drugs, the cost of producing new drugs can be reduced. For the enterprise, it also saves materials and is conducive to its sustainable development. A comparison chart of the two in terms of corporate earnings is shown in Figure 9.

Through the comparison of Figure 9, it was found that the income based on blockchain was higher than that of reverse logistics at the current stage. Through the comparison of the overall income of the two quarters, it was found that the increase in interest was about 19.5%.

## 5. Conclusions

The focus of this paper is to propose the system architecture, working mechanism, and development characteristics of blockchain technology. It solves the problems of clarity of reverse logistics at the current stage, as well as the instability of the system, the complexity of operations, the complexity of goal realization, the repetition of operations, and the repetition of task completion. Taking advantage of the technical characteristics of blockchain and the cross-connection between it and the clarity of reverse logistics, a reverse logistics information system model developed from the perspective of blockchain has been given. Furthermore, the working principle of this information system model was expounded. By comparing with the current green reverse engineering logistics products, building a model through the technical mode of blockchain and the framework of information utilization, the functional principle of the information system model was expounded. After comparing the reverse logistics methods of various enterprises at this stage, it is believed that the adoption of the enterprise reverse logistics information system model under the blockchain can make organic integration between different links in the entire supply chain. Therefore, the operation process of reverse logistics of modern enterprises can be greatly improved, thereby reducing the logistics costs of traditional enterprises and saving the human resources of the whole society. The disadvantage of this paper is that it does not elaborate on blockchain technology and does not explain the details of reverse logistics, such as recycling routes. It is expected that under the future technology, the current reverse logistics system will be more and more complete, with a huge impact on the environment, companies, and individuals.

The article "Sustainable Development of Green Reverse Logistics Based on Blockchain" was retracted in 2023. Reasons: signs of a paper mill; suspected computer-generated content; unreliable results or conclusions; lack of ethics approval or compliance.

## Figures and Tables

**Figure 1:** Significance of “green reverse logistics.”

**Figure 2:** Important pathways to sustainable development.

**Figure 3:** Main factors of green reverse logistics.

**Figure 4:** Drug recall process.

**Figure 5:** Reverse logistics network model under a random drug defect level.

**Figure 6:** Comparison of recycling efficiency.

**Figure 7:** Comparison of scrap rates.

**Figure 8:** Comparison of utilization.

**Figure 9:** Comparison of corporate earnings.

**Table 1:** Relevant technical directions in the field of reverse logistics.

Relevant technologies in the field of reverse logistics and method	Companies should be encouraged to improve product design	Advances in resource recycling technology	New energy-saving technology
1	Improve product quality	Waste recycling	Use clean energy
2	Improve product quality	Develop reverse logistics	Use environmentally friendly vehicles
3	Promote green packaging	—	Purification of waste gas and wastewater

## Data Availability

The data that support the findings of this study are available from the corresponding author upon reasonable request.
